# HSPB8 Overexpression Ameliorates Cognitive Impairment in Diabetic Mice via Inhibiting NLRP3 Inflammation Activation

**DOI:** 10.1155/2022/9251835

**Published:** 2022-08-01

**Authors:** Yanmin Chang, Yanqing Wu, Xingjun Jiang, Jiahui Zhu, Cailin Wang, Rong Ma, Gang Li

**Affiliations:** ^1^Department of Neurology, Union Hospital, Tongji Medical College, Huazhong University of Science and Technology, Wuhan, China; ^2^Department of Pharmacology, Tongji Medical College, Huazhong University of Science and Technology, Wuhan, China

## Abstract

Type 2 diabetes mellitus (T2DM) is associated with an elevated risk of cognitive impairment. And the underlying mechanism remains unillustrated. HSPB8 is a member of the small heat shock protein family. In this study, we found that the expression of HSPB8 was upregulated in the hippocampus of high − fat diet (HFD) + streptozotocin (STZ) −  induced diabetic mice and N2a cells exposed to high glucose. Overexpression of HSPB8 relieved cognitive decline in DM mice. Mechanically, HSPB8 overexpression in the hippocampus of diabetic mice inhibited NOD-like receptor protein 3 (NLRP3) inflammasome activation via dephosphorylating mitochondrial fission-associated protein dynamin-related protein 1 (DRP1) at the phosphorylated site Ser616 (p-Drp1S616). Furthermore, HSPB8 overexpression increased mitochondrial membrane potential (MMP) and reduced oxidative stress. These results indicate a protective effect of HSPB8 in the hippocampus of diabetic mice and N2a cells exposed to high glucose. Overexpression of HSPB8 might be a useful strategy for treating T2DM-related cognitive decline.

## 1. Introduction

Diabetes mellitus is a common metabolic disorder that can cause multiple comorbidities, such as nephropathy, cardiovascular disease, and retinopathy [1]. Additionally, people with type 2 diabetes mellitus perform poorly on learning and memory tests [2]. Due to the diabetes pandemic and the concomitant rise in the aging population worldwide, diabetes-related cognitive dysfunction substantially affects society and seriously affects patients' quality of life and has received significant attention [3]. But the potential mechanisms underlying Type 2 diabetes mellitus (T2DM) related cognitive decline remain elusive. Therefore, it is urgent to clarify the pathogenesis of diabetes-related cognitive decline and find effective prevention and treatment strategies.

HSPB8, Heat shock protein 22 (HSP22), known as H11 kinase, E21G1, is a member of the small HSP family of proteins containing an *α*-crystalline domain and has been demonstrated to have a protective effect against various conditions including oxidative stress, aging, cancer, and apoptosis [4–7]. Notably, HSPB8 could regulate mitochondrial biogenesis and prevent excessive mitochondrial fission [5].

Mitochondria are dynamic organelles providing necessary energy for cells. The morphology of these organelles can make adaptive changes according to the needs of the cells and undergo continuous fusion and fission. Mitochondrial fusion and fission defects would cause mitochondrial dysfunction [8–10]. Mitochondrial fusion is mainly mediated by the fusion proteins Mfn1, Mfn2, and OPA1 [11, 12]. The central player in mitochondrial fission is DRP1 [13]. The activity of DRP1 is mediated by phosphorylation of two critical phosphorylation sites, serine 616 (active form) and serine 637 (inactive form) [8, 10, 14, 15]. Due to the vital role of mitochondria homeostasis in the T2DM-related cognitive decline, it is vital to explore whether overexpression of HSPB8 could ameliorate mitochondrial dysfunction in the brains of the T2DM mouse model.

In the current study, we used mice treated with a high-fat diet and streptozotocin to mimic T2DM. The results showed upregulated expression of HSPB8 in the hippocampus of diabetic mice and N2a cells exposed to high glucose. Overexpressing HSPB8 in the hippocampi inhibited NLRP3 inflammasome activation via dephosphorylating DRP1 at the phosphorylated site Ser616 (p-Drp1S616), reduced oxidative stress, and ultimately relieved cognitive impairments. This study suggests that HSPB8 could be a promising therapeutic target for T2DM-related cognitive decline.

## 2. Materials and Methods

### 2.1. Animals

Male C57BL/6 mice (7-week-old) were purchased from Beijing Vital River Laboratory Animal Technology Co., Ltd. These mice were randomly divided into four groups (*n* = 20 per group). Two groups of mice were fed with high-fat diet (HFD) (60 kcal% fat). Then, at 20 weeks old, mice were treated with streptozotocin (STZ) (100 mg/kg) by intraperitoneal (i.p.) injection. One week later, we detected blood glucose levels with fasting 12 h. Mice with the features (polyphagia, polydipsia, and polyuria) and blood glucose levels exceeding 11.1 mmol/L were thought to be T2DM. At 28^th^ week, the virus was injected into the hippocampus. One group of mice received virus AAV-HSPB8-EGFP (group: DM + HSPB8). Another group received the control virus AAV-EGFP (group: DM). Another two groups of mice were treated with normal diet. Then, mice received a single dose of citrate buffer vehicle (pH 4.5). One group of mice received virus AAV-HSPB8-EGFP(group: WT + HSPB8). Another group received the control virus AAV-EGFP (group: WT). All animals were housed in a specific pathogen-free environment at 22°C, with 12 h light-dark cycles. Mice were allowed to move for food and water freely. Animal experiments were performed according to protocols approved by the animal ethics committee of Tongji Medical College, Huazhong University of Science and Technology.

### 2.2. Stereotactic Injection

Adeno-associated virus was coded for HSPB8 with enhanced green fluorescent protein EGFP. AAV-HSPB8-EGFP (1 × 10^13^ vg/mL) and the control AAV-EGFP (1 × 10^13^ vg/mL) were obtained from OBiO Biologic Technology Co., Ltd. (Shanghai, China). Mouse was fixed on stereotaxic apparatus after anesthesia with isoflurane. Animals were bilaterally injected with 1 *μ*L of virus into the hippocampus (AP-1.9 mm; ML ± 1.5 mm; DV-1.9 mm) at an injection rate of 100 nl/min. Before being removed, the needle was allowed to remain for an additional 10 min. Behavioral tests were performed 4 weeks after virus injection.

### 2.3. Novel Object Recognition (NOR)

According to the previous report [16], a novel object recognition test was performed in a box (50 × 50 × 50 cm). First, mouse was put in the box to adapt to the environment for 5 min in an empty box 24 h before testing. Two identical objects (A and B) were put at two different corners during the training phase. Mice were placed in the center of the bottom and allowed to explore for 5 min freely. Time to explore each object was recorded. Twenty-four hours later, the testing phase began. A differently new object C was used to take the place of object A. And mice were placed in the box to explore for another 5 min. Time to explore object B and object C was recorded. The recognition index was calculated as (object C exploration time)/(object A exploration time + object C exploration time).

### 2.4. Morris Water Maze (MWM)

Morris water maze test was carried out to evaluate spatial learning and memory. A circular pool (120 cm diameter) filled with water was divided into 4 quadrants. 1.5 cm beneath the water surface, a platform (10 cm diameter) was placed in a fixed position at the center of the target quadrant. The mice were trained to find the platform for five consecutive days. Mice were put into water from four different quadrants daily for 60 s or till the platform was found and then they were allowed to rest on the platform for 20 s. Latencies loading to the platform were recorded. After 24 h of the last training, a probe test was conducted. In the probe test, the platform was removed and the number of times the mice crossed through the platform position, and the time stayed at the target quadrant and the locus of the movement was recorded (60 s of test duration). All data were recorded by using Chengdu Taimeng Software Co. Ltd. (China).

### 2.5. Western Blotting

Protein samples from all groups were lysed with RIPA lysis buffer. Via centrifugation at 12,000 g for 15 min at 4°C, the supernatant was obtained. Protein concentration was decided by the BCA Protein Assay kit (Beyotime, Shanghai, China). After SDS acrylamide gel electrophoresis, the proteins were subjected to transfer onto nitrocellulose membranes (Amersham Biosciences, Germany). Following by blocking with 5% BSA at 25°C for 1 h, the membranes were incubated with primary antibodies overnight at 4°C. Primary antibodies used were listed in Table 1. After that, the membranes were subjected to incubation with the corresponding secondary antibody for 1 h at room temperature. Finally, the proteins were visualized by Odyssey Infrared Imaging System (Licor biosciences, Lincoln, NE, USA) and ECL Imaging System (610007-8Q, Clinx Science Instruments Co., Ltd.). The quantitative analysis of proteins was performed by using ImageJ software.

### 2.6. Golgi Staining

Golgi staining was conducted using FD Rapid GolgiStainTM kit (FD NeuroTechnologies, USA). Hippocampus from all groups was immersed in solutions A and B at room temperature for 4 weeks. After that, brains were transferred into solution C in the dark for a week. Brain tissues were sliced at a thickness of 100 *μ*m. The slices were stained in a mixture of solution D and solution E for 10 min. Following dehydrating with ethanol and clearing with xylene, the sections were mounted on slides.

### 2.7. Immunofluorescence

Brains were paraffin-embedded, and slices (5 *μ*m thickness) were used for immunofluorescence analysis. After removing paraffin with xylene, slices were subjected to rehydrated through incubation in gradient ethanol. Followed by antigen repairing in sodium citrate, the slices were then going through membrane rupturing with 0.5% Triton X-100 and blocking in 5% BSA at room temperature. After that, sections were incubated with primary antibodies at 4°C overnight. The primary antibodies were as follows: after 3 times washing with PBS, sections were incubated with fluorescent secondary antibodies (Alexa Fluor 488 and 594). DAPI was needed for the staining of nuclei for 10 min at 25°C. Finally, immunofluorescence images were observed with a microscope (SV120, OLYMPUS).

### 2.8. Quantitative Real-Time PCR

Total RNA was extracted from hippocampi of all groups using Trizol reagent (TaKaRa). The reverse transcription and amplification were performed according to manufacturer's instruction (TaKaRa). RT-PCR was conducted on a StepOne Plus Real-Time PCR Detection System (Applied Biosystems). The expression level of the target gene was normalized to *β*-actin mRNA expression level and calculated by the 2*ΔΔ*Ct method for relative expression analysis. Primers employed in this study were listed in Table 2.

### 2.9. Transmission Electron Microscopy

Hippocampi were separated and fixed in 2.5% glutaraldehyde at 4°C. Then, tissues were postfixed with 1% osmium tetroxide for 2 h. After that, samples were subjected to dehydrate in graded ethanol and followed by embedding in epoxy resin. The tissues were cut into ultrathin sections (50 nm). After staining with uranyl acetate for 20 min and lead citrate for 5 min, slices were observed with a transmission electron microscope (Thermo Fisher Scientific).

### 2.10. SOD, CAT, and MDA Assays

To detect superoxide dismutase (SOD), catalase (CAT), and malondialdehyde (MDA), mice were anesthetized and decapitated. Hippocampus was rapidly removed and homogenized. After centrifugation, the supernatant was collected to evaluate the levels of MDA (Beyotime, Haimen, China) and activities of SOD (Nanjing Jiancheng Bioengineering Institute, Nanjing, China) and CAT with assay kits (Nanjing Jiancheng Bioengineering Institute, Nanjing, China) following the manufacturer's directions.

### 2.11. Cell Culture, Treatments, and Transfection

Mouse N2a neuroblastoma cells were obtained from Professor Gongping Liu from Tongji Medical College, Huazhong University of Science and Technology. Cells were cultured in Dulbecco's modified Eagle's medium (containing 25 mM glucose, NG group) supplemented with 10% FBS, streptomycin/penicillin (1%). When cells were approximately 70–80% confluent, they were exposed to high glucose condition (HG group). In the present study, 100 mM concentration of glucose was used as high glucose condition [17]. For transfection experiments, N2a cells were plated onto 12-well plates, and HSPB8-EGFP plasmids (OBiO Biologic Technology, Shanghai) and shRNA(HSPB8)-EGFP (OBiO Biologic Technology, Shanghai) were transfected using NEOFECTTM DNA transfection reagent (NEOFECT, Beijing). All cells were maintained in a humidified incubator at 37°C under 5% CO_2_ containing atmosphere.

### 2.12. Assessment of Mitochondrial Membrane Potential by JC-1

The mitochondrial membrane potential (MMP) was measured by JC-1 dye (Beyotime, Haimen, China). N2A cells were incubated with cell culture medium mixed with JC-1 staining working solution and mixed well. After incubation at 37°C for 20 minutes, the supernatant was removed and washed cells twice with JC-1 staining buffer. Then, add 2 mL fresh medium to the well.

Finally, cells were observed under confocal microscope (Leica, Germany). The ratio of red and green fluorescence was analyzed.

### 2.13. Statistical Analysis

Data were expressed as the Mean ± SEM. Statistical analysis was performed using GraphPad Prism 9. Comparisons were evaluated using unpaired Student's *t*-test, one-way ANOVA, or two-way repeated measures ANOVA followed by Tukey's post hoc test. Differences with *p* < 0.05 were considered as statistical significance.

## 3. Results

### 3.1. Increased HSPB8 Protein Expression in the Hippocampus of DM Mice

We measured the protein (Figures 1(a) and 1(b)) and mRNA levels (Figure 1(c)) of HSPB8 in the hippocampus of WT and DM mice. Upregulation of HSPB8 was detected in DM mice. These findings were validated by immunofluorescence staining (Figure 1(d)). Overexpression of HSPB8 was shown by western blotting and immunofluorescence in the virus-injected hippocampus (Figure 1(e) and 1(f)).

### 3.2. HSPB8 Overexpression Relieves Cognitive Dysfunction in DM Mice

To explore the role of HSPB8 overexpression in learning and memory abilities, we conducted the Morris water maze (MWM) and novel object recognition (NOR) tests. In the MWM test, DM mice showed longer latency to reach the platform during the training stage, indicating memory deficits than WT mice. However, HSPB8 overexpression attenuated the spatial learning deficits, as shown by the downregulated escape latency at the 4th and 5th day during the training phase (Figure 2(a)). On the 7th day, by removing the platform, we found that HSPB8 overexpression ameliorated the DM mice's memory deficits as they spent less time arriving platform placed previously (Figure 2(b)), increased time stayed in the target quadrant (Figure 2(c)), and the times across the target quadrant (Figure 2(e)). A representative swimming trace was shown (Figure 2(d)). No significant difference in swimming speed was detected (Figure 2(f)), indicating no motor dysfunction among the four groups. Furthermore, NOR was performed, and DM mice spent less time with the novel object compared with WT mice, which indicated cognitive impairment. While HSPB8 overexpression ameliorated this performance, showing upregulated time spent with the new novel object at 24 h in DM mice (Figure 2(g)).

These results suggest that HSPB8 overexpression relieved cognitive dysfunction in DM mice.

### 3.3. HSPB8 Overexpression Relieves Synaptic Damages in DM Mice

Golgi staining was performed to reveal the change of density of the spine in the hippocampus.

We observed a reduction in spine density in the DM group when compared with the WT group.

Then, HSPB8 overexpression ameliorated the decrease of spine density in DM mice (Figures 3(a) and 3(b)). Furthermore, we performed transmission electron microscopy. The result showed a significant synapse loss in the hippocampus of DM group when compared with the WT group. Notably, HSPB8 overexpression increased the number of synapses in the hippocampus of DM mice (Figures 3(c) and 3(d)). These data suggest that HSPB8 overexpression relieved synaptic damages in DM mice.

### 3.4. HSPB8 Overexpression in the Hippocampus Alleviates Mitochondrial Fission

Mitochondria are highly dynamic organelles, continuously going through fission and fusion. Dynein-related protein 1 (DRP1) is a critical regulator resulting in mitochondrial fission. We did not detect a significant increase in DRP1 expression in the hippocampus of DM group compared to WT group. However, the result of western blotting showed that p-Drp1/Drp1 was upregulated (Figures 4(a) and 4(b)). The levels of p-Drp1 were also upregulated in the hippocampus of DM group compared with WT group, as shown by immunostaining (Figure 4(c)). After HSPB8 overexpression, western blotting and immunostaining showed decreased expression levels of p-Drp1/Drp1 (Figures 4(a)–4(c)). In addition, we examined the levels of mitochondrial fusion proteins Mitofusin-1 (MFN1), Mitofusin-1 (MFN2), and optic atrophy1 (OPA1) by western blot. As shown in Figures 4(a) and 4(b), the levels of MFN1 and MFN2 were reduced in DM group compared to WT group. However, HSPB8 overexpression did not affect their expression. Electron microscopy revealed that the size of mitochondria in the hippocampus of the DM group was decreased compared to the WT group (Figure 4(d)). HSPB8 overexpression decreased the number but increased the length of the mitochondrial in DM + HSPB8 group compared with DM group (Figures 4(f) and 4(g)).

### 3.5. HSPB8 Overexpression in the Hippocampus Alleviates Oxidative Stress

Next, due to the important role of oxidative stress (OS) in the T2DM-related cognitive decline, we explored the role of HSPB8 on OS. As shown in Figures 5(a) and 5(b), the activity of superoxide dismutase 1 (SOD) and catalase (CAT) was reduced in the hippocampus of DM group compared with WT group. Malondialdehyde (MDA), used to assess lipid peroxidation, was significantly elevated in DM mice (Figure 5(a)). HSPB8 overexpression reversed the pathological changes in DM mice. Western blotting revealed the same results that protein levels of critical antioxidant enzymes SOD1 and CAT were significantly declined in the DM mice compared with WT mice (Figures 5(d)–5(f)). Moreover, HSPB8 overexpression increased the expression of SOD1 and CAT in the hippocampus of DM mice.

Taken together, our findings revealed that HSPB8 could alleviate oxidative stress.

### 3.6. HSPB8 Overexpression in the Hippocampus Alleviates NLRP3 Inflammation in DM Mice

In this study, we also evaluated the effect of NLRP3 in DM mice. NLRP3 inflammasome signals, including NLRP3, ASC (apoptosis-associated speck-like protein), cleaved caspase1 p20, and IL-1*β* (interleukin-1*β*), were measured by western blotting, as shown in Figures 6(a)–6(e).

NLRP3, ASC, cleaved caspase1 p20, and IL-1*β* were upregulated in the hippocampus of the DM mice compared with WT mice. However, HSPB8 overexpressing reversed these changes (Figures 6(a)–6(e)).

These results suggest that HSPB8 overexpression inhibits NLRP3 inflammasome activation in DM mice.

### 3.7. HSPB8 Overexpression Attenuates MMP and NLRP3 Inflammasome Activation in High Glucose-Treated N2a Cells

The protein level of HSPB8 was significantly upregulated in high glucose-treated cells when compared with exposed to normal glucose (NG) (Figure 7(a)). Mitochondrial membrane potential (MMP) was measured by JC-1 staining. High glucose treatment decreased the MMP in N2a cells compared with cells treated with NG, while overexpression of HSPB8 and mdivi-1 treatment reversed high glucose-mediated downregulation of MMP (Figures 7(b) and 7(c)). In addition, we evaluated the effect of HSPB8 on DRP1 at S616 phosphorylation in N2a cells (Figures 7(d) and 7(e)). HSPB8 overexpression and Mdivi-1 treatment decreased the ratio of p-Drp1/Drp1 (Figure 7(a)). In the meantime, the protein levels of NLRP3, cleaved caspase1 p20, ASC, and IL-1*β* were also decreased (Figures 7(f)–7(i)).

These results suggest that HSPB8 overexpression attenuates MMP and NLRP3 inflammasome activation in HG-treated N2a cells via inhibiting mitochondrial fission.

## 4. Discussion

In this study, we report elevated expression of HSPB8 in the hippocampus of diabetic mice and the N2a cells exposed to high glucose. The heat shock family is composed of many proteins which are induced by various stress. HSPB8 is a kind of small heat shock protein [18]. Our result is consistent with previous experimental studies showing upregulated protein levels of HSPB8 under various stress. According to the previous reports, it exacted beneficial effect on alleviating mitochondrial biogenesis, oxidative stress, endothelial cell activation, and reduced apoptosis [4–7]. HSPB8 is mainly regulated by heat shock factor signaling; however, it was prevented from further increasing due to a negative feedback loop between the heat shock factor and HSPB8. Thus, HSPB8 cannot constantly increase and fully exert its effects under stress [7, 19]. The current study demonstrated that overexpression of HSPB8 exacted protective effects, which in turn ameliorated the excessive mitochondrial fission, aggravated neuroinflammation, reduced oxidative stress, and ultimately relieved cognitive impairments.

Mitochondria are highly dynamic organelles that continuously change their size, shape, and numbers via fusion and fission to supply the energy required for the cells and maintain metabolic homeostasis [8, 20]. An increasing number of studies suggested that Dynein-related protein 1 (DRP1) is a critical regulator in mitochondrial fission. Protein phosphorylation is a posttranslational modification. It is widely used to regulate protein functions in cells. The phosphorylation residue of p-Drp1S616 was a vital residue for regulating DRP1. Increasing p-Drp1S616 showed extended phosphorylation of DRP1 and induced excessive mitochondrial fission [21–23]. In this study, evidence showed that the expression of p-Drp1S616 was upregulated in the hippocampus of DM mice. Our finding is consistent with the results that the expression of p-Drp1S616 in the hippocampus of leptin-deficient (ob/ob) was elevated [24]. In the hippocampus of DM mice, transmission electron microscopy demonstrated that mitochondrial number was increased, and length was decreased compared with WT mice. Conversely, overexpression of HspB8 could downregulate the number and increase the length of mitochondria. p-Drp1S616 was increased in N2a cells exposed to high glucose. These findings are consistent with the in vivo results. In addition, JC-1 was performed to investigate mitochondrial membrane potential (MMP). High glucose exposed N2a cells showed decreased MMP. HSPB8 overexpression inhibited high glucose-induced loss of membrane potential.

Hippocampus is rich in mitochondria and generates energy for synaptic activity. Mitochondrial dynamics are impaired in the hippocampus of diabetic mice [25], which results in reducing energy metabolism, disrupting cell signal cascade, and ultimately causing synaptic damage and cognitive dysfunction [26–28]. In the present study, the DM mice displayed excessive mitochondrial fission. Abnormal mitochondrial dynamics may contribute to neuronal damage leading to lack of ATP energy in the hippocampus. These findings indicated that HSPB8 might ameliorate synaptic damage and cognitive dysfunction in diabetic mice due to regulating mitochondrial fission. Furthermore, the expression levels of MFN1, MFN2, and OPA1 were decreased. However, HSPB8 overexpression did not change their levels in DM mice, indicating that HSPB8 may not be able to regulate mitochondrial fusion, or we need more samples to explore the effect.

Oxidative stress (OS) plays a crucial role in the pathogenesis of various neurodegenerative diseases [29, 30]. It could reduce the production of ATP, which is critical for neuron survival and metabolism. Therefore, OS is acknowledged as a key factor in the deterioration of learning and memory in the hippocampus [31–33]. In this study, we explored several certain biochemical parameters such as SOD, MDA, and catalase. Results showed decreased activity of SOD and catalase and elevated levels of MDA in the hippocampus of DM mice compared with WT mice. HSPB8 overexpression reversed described levels for cognitive decline. Additionally, the western blotting of SOD1 and catalase showed consistent results. As antioxidant enzyme, SOD1 and catalase were reduced in DM mice compared with WT mice, leading to a subsequent increase in oxidative stress. HSPB8 overexpression suggested an ameliorative antioxidative capacity in the hippocampus of DM mice. HSPB8 overexpression helped to mediate the oxidative stress system and improved cognitive impairment. These results concordant with previous findings that HSPB8 overexpression protects cells from oxidative stress [6, 7].

NLRP3 inflammasome activation is known to contribute to diabetes and dementia by triggering IL-1*β* maturation. NLRP3 inflammasome activation was also observed in diabetic cognitive impairment model mice/rats [34, 35]. Mitochondrial fission was reported to regulate NLRP3 inflammasome activation [36–38]. Further experiments in vitro revealed that when the ratio of p-Drp1S616/DRP1 was upregulation, the activation of NLRP3 inflammasomes, including NLRP3, cle-caspase-1, and IL-1*β* was increased. HSPB8 overexpression or treatment with Mdivi-1 (a specific inhibitor of Drp1) inhibited DRP1 phosphorylation at Ser-616 and thus reduced excessive mitochondrial fission in N2a cells exposed to high glucose. This result is consistent with previous studies that mdivi-1 exacted the protection by decreasing phosphorylation of DRP1 at serine 616 (p-Drp1S616) [39–41]. It is reported that exogenous HSPB8 significantly conveys neuroprotection via attenuation of mitochondrial damage partly by suppressed drp1-mediated mitochondrial fission through AMPK-PGC1*α* signaling pathway after subarachnoid hemorrhage (SAH). Whereas knockdown of HSPB8 reversed the above protective effects [5]. According to the above, HSBP8 should be the upstream cause of downregulation of p-Drp1S616. Importantly, we observed that the activation of NLRP3 inflammasomes was downregulated after treatment with HSPB8 or mdivi-1. Mdivi-1 attenuated activation of NLRP3 inflammasomes by downregulating mitochondrial fission in N2a cells exposed to high glucose. At the same time, mdivi-1 treatment did not affect the expression of HSPB8. On the contrary, knocking down the expression of HSPB8 elevated the levels of p-Drp1/Drp1, NLRP3, cleaved caspase-1 p20, and IL-1*β*. Collectively, the available evidence indicated that HSPB8 could downregulate mitochondrial fission, thus suppress the activation of NLRP3 inflammasome. Our findings confirm that regulation of mitochondrial dynamics could be a new therapeutic alternative for diabetic complications [25]. At the same time, we provide a new possibility for the activation of NLRP3.

## 5. Conclusions

In the present study, we revealed elevated expression of HSPB8 protein in the hippocampus of diabetic mice. Overexpressing HSPB8 in the hippocampi could inhibit NLRP3 inflammasome activation via regulation of Drp1 phosphorylation (p-Drp1S616), reduce oxidative stress, and relieve cognitive impairments in diabetic mice. These results suggest that HSPB8 could be a promising therapeutic target for Type 2 diabetes mellitus(T2DM)-related cognitive decline.

## Figures and Tables

**Figure 1:** Upregulation of HSPB8 in the hippocampus of DM mice. (a, b) Representative western blot images and quantitative analyses of HSPB8 in the hippocampus of WT and DM mice (*n* = 5 mice per group). ^∗∗^, *p* < 0.01. (c) mRNA levels of HSPB8 in the hippocampus of WT and DM mice were detected by PCR. ^∗∗^, *p* < 0.01. (d) Representative immunofluorescence staining images of HSPB8 (red) in the hippocampus of WT and DM mice. Nuclei were counterstained with DAPI (blue). Scale bar = 200 *μ*m. (e) Upregulation of HSPB8 was confirmed by western blotting and (f) immunofluorescent staining when injected virus in the hippocampus (*n* = 5 mice per group).

**Figure 2:** Overexpression of HSPB8 relieved cognitive dysfunction in DM mice. (a) Latency to the platform during training stage in Morris water maze (MWM), *n* = 11 mice/group, two-way repeated-measures ANOVA test followed by Tukey's post hoc test, ^∗^, *p* < 0.05, ^∗∗∗^, *p* < 0.001, ^∗∗∗∗^, *p* < 0.0001, WT group vs. DM group; ^#^*p* < 0.05, DM group vs. DM + HSPB8 group. (b–f) The cognitive ability was detected by MWM. (b) Escape latency, (c) time in the target quadrant, (d) the representative swimming path of the mice during the MWM probe test, (e) and times across the platform. (f) There was no significant difference in swimming speed among the four groups. (*n* = 10 − 13 mice/group). ^∗^, *p* < 0.05, ^∗∗^, *p* < 0.01. (g) Recognition index during training and test in new object recognition (NOR) (*n* = 10 mice/group). ^∗^, *p* < 0.05, ^∗∗^, *p* < 0.01.

**Figure 3:** Overexpression of HSPB8 relieved synaptic damages in DM mice. (a, b) Dendritic spine density was detected by Golgi staining in the hippocampal regions and quantitative analysis. Scale Bar, 10 *μ*m. (*n* = 3 mice per group). (c, d) The synaptic density in the hippocampus of mice was detected by electron microscopy and quantitative analysis (*n* = 3 mice for each group). Blue arrows indicate synapses. Scale bar = 2 *μ*m. All data are shown as the mean ± SEM. One-way ANOVA test followed by Tukey's post hoc test, ^∗^*p* < 0.05, ^∗∗∗^, *p* < 0.001.

**Figure 4:** HSPB8 overexpression in the hippocampus alleviates mitochondrial fission. (a) Expressions of p-Drp1, Drp1, MFN1, MFN2, and OPA1 in the hippocampus were detected by Western blot. *β*-Actin was used as loading control. (*n* = 5 each group) and (b) quantitative analysis. ^∗^, *p* < 0.05, ^∗∗^, *p* < 0.01, ^∗∗∗∗^, *p* < 0.0001. (c, d) Representative images of immunofluorescence staining against p-Drp1 (green) in the (dentate gyrus) DG and CA1. Nuclei were counterstained with DAPI (blue) (*n* = 3 mice per group). Scale bar = 100 *μ*m. (e) Representative electron microscopy images showing mitochondrial morphology in hippocampal neurons (*n* = 3 mice per group). Scale bar = 1 *μ*m. (f, g) Measurements of mitochondrial numbers and mitochondrial length. One-way ANOVA test followed by Tukey's post hoc test. Data are shown as the mean ± SEM. ^∗^*p* < 0.05, ^∗∗^, *p* < 0.01.

**Figure 5:** HSPB8 overexpression in the hippocampus alleviates oxidative stress. (a–c) The superoxide dismutase (SOD), catalase (CAT), and malondialdehyde (MDA) levels in the hippocampus of four groups (*n* = 3 mice per group). (d–f) Western blotting and quantification of SOD1 and CAT in the hippocampus (*n* = 5 mice per group). *β*-Actin was used as loading control. All data are shown as the mean ± SEM. One-way ANOVA test followed by Tukey's post hoc test, ^∗^*p* < 0.05, ^∗∗^, *p* < 0.01, ^∗∗∗^, *p* < 0.001, ^∗∗∗∗^, *p* < 0.0001.

**Figure 6:** HSPB8 overexpression in the hippocampus alleviates NLRP3 inflammation in DM mice. (a–e) Western blotting and quantification of NLRP3, ASC, caspase-1 p20, and IL-1*β* levels in the hippocampus of four groups of mice (*n* = 5 each group). *β*-Actin was used as loading control. All data are shown as the mean ± SEM. One-way ANOVA test followed by Tukey's post hoc test, ^∗^*p* < 0.05, ^∗∗^, *p* < 0.01, ^∗∗∗^, *p* < 0.001.

**Figure 7:** Overexpression of HSPB8 attenuates MMP and NLRP3 inflammasome activation in high glucose treated N2a cells. (a) Representative western blot images and quantitative analyses of HSPB8 in cells from all groups. *β*-Actin was used as loading control. (b) Representative images of JC-1 immunochemistry staining showing the mitochondrial membrane potential in each group of cells. (c) Relative quantitative comparison of red-to-green fluorescence intensity ratios between each group. (d–i) Expressions of p-Drp1, Drp1, NLRP3, cleaved caspase1 p20, and IL-1*β* in N2A cells of all groups were detected by western blot and quantitative analysis. *β*-Actin was used as loading control. All data are shown as the mean ± SEM. Two-tailed Student's *t*-test, ^∗^*p* < 0.05, ^∗∗^, *p* < 0.01, ^∗∗∗^, *p* < 0.001, ^∗∗∗∗^, *p* < 0.0001.

**Table 1:** Antibodies used in this study.

Antibody	Host	Dilution (WB)	Dilution (IF)	Company
Anti-HSPB8	Rabbit	1 : 500	1 : 50	Abcam
Anti-*β*-actin	Mouse	1 : 4000		Proteintech
Anti-NLRP3	Rabbit	1 : 1000		Abcam
Anti-Caspase1	Rabbit	1 : 1000		Proteintech
Anti-IL-1*β*	Rabbit	1 : 1000		Proteintech
Anti-ASC	Mouse	1 : 1000		Santa Cruz
Anti-MFN1	Rabbit	1 : 1000		Cell Signaling Technology
Anti-MFN2	Rabbit	1 : 1000		Cell Signaling Technology
Anti-OPA1	Rabbit	1 : 1000		ABclonal
Anti-DRP1	Rabbit	1 : 1000		ABclonal
Anti-(pDrp1S616)	Rabbit	1 : 1000	1 : 50	ABclonal
Anti- SOD1	Rabbit	1 : 1000		Proteintech
Anti-catalase	Rabbit	1 : 1000		ABclonal

**Table 2:** 

Gene	Forward primer (5′ to 3′)	Reverse primer (5′ to 3′)
HSPB8	ATGAAGAGAAGC AGCAGGAAGGTG	TGGTTGTCTTGA GGAAGCTCGTTG
*β*-Actin	GGCTGTATTCCC CTCCATCG	CCAGTTGGTAAC AATGCCATGT

## Data Availability

The data sets used for the current study are available from the corresponding author upon reasonable request.

## Abbreviations

STZ: Streptozotocin
HFD: High-fat diet
NOR: Novel object recognition
MWM: Morris water maze
WB: Western blot
MMP: Mitochondrial membrane potential
OS: Oxidative stress
HSP: Heat shock proteins
SOD: Superoxide dismutase
CAT: Catalase
MDA: Malondialdehyde.
